The article "Value of Postoperative Serum Albumin to Predict Postoperative Complication Severity in Spinal Tuberculosis" was published in 2022. Journal: Biomed Res Int.

# Value of Postoperative Serum Albumin to Predict Postoperative Complication Severity in Spinal Tuberculosis

**DOI:** 10.1155/2022/4946848

**Published:** 2022-02-09

**Authors:** Guanyin Jiang, Xing Du, Yong Zhu, Muzi Zhang, Wanyuan Qin, Tuotuo Xiong, Yunsheng Ou

**Affiliations:** Department of Orthopedics, First Affiliated Hospital of Chongqing Medical University, Chongqing 400016, China

## Abstract

**Background:**

Many complications occur after surgery in patients with spinal tuberculosis (STB); however, the severity varies in different patients. The complications' severity is evaluated from grades I to V by the Clavien–Dindo classification (CDC), and grade V is the most severe. Most complications are mild, and only severe complications are life threatening, and thus, it is important to identify severe complications in patients with STB. The purpose of this study was to identify the risk factors of postoperative complication severity in patients with STB.

**Methods:**

Between January 2012 and May 2021, a retrospective study included 188 patients that underwent STB debridement surgery. The patients were divided into three groups based on postoperative complication severity. Clinical characteristics measured included age, sex, body mass index (BMI), comorbidities of diabetes mellitus and pulmonary tuberculosis, alcohol use and smoking history, course of disease, preoperative hemoglobin, preoperative serum albumin, preoperative lymphocytes, preoperative erythrocyte sedimentation rate (ESR), preoperative C-reactive protein (CRP), surgical approach, operating time, blood loss during surgery, postoperative hemoglobin, and postoperative serum albumin. The clinical characteristics of patients with STB who developed postoperative complications were evaluated using logistic regression analysis.

**Results:**

188 patients suffered at least one postoperative complication; 77, 91, and 20 patients experienced grade I, II, and III-IV complications, respectively. In the univariate analysis, sex, diabetes mellitus, postoperative hemoglobin, and postoperative albumin are statistically significant. In the multivariable analysis, postoperative albumin (adjusted odds ratio (OR) = 0.861, *P* < 0.001) was an independent risk factor of the postoperative complication severity in patients with STB. Receiver operating characteristic (ROC) analysis showed that the optimal cutoff values for postoperative albumin were 32 g/L (sensitivity: 0.571, specificity: 0.714, area under the ROC curve: 0.680) and 30 g/L (sensitivity: 0.649, specificity: 0.800, area under the ROC curve: 0.697) for grade II and grade III-IV complications, respectively.

**Conclusions:**

Postoperative albumin is an independent risk factor for postoperative complication severity in patients with STB. The improvement of postoperative albumin levels may reduce the risk of severe complications in patients with STB.

The article "Value of Postoperative Serum Albumin to Predict Postoperative Complication Severity in Spinal Tuberculosis" was published in 2022. Journal: Biomed Res Int.

## 1. Introduction

Spinal tuberculosis (STB) is a type of osteoarticular tuberculosis with high morbidity, taking part of 50% in osteoarticular tuberculosis [1]. Standard antituberculosis (TB) drug administration combined with timely surgery is an important and effective treatment for patients with STB [2]. Lesion focus debridement is a significant treatment in STB therapy, which enhances tuberculosis control, promotes bone graft fusion, improves the efficacy of antituberculosis drugs, and reduces the risk of STB recurrence [3, 4]. However, debridement of the spinal focus is an iatrogenic trauma that usually causes considerable blood loss. In addition, most patients with STB have comorbidities, such as diabetes, anemia, and hypoalbuminemia, and thus, they are susceptible to the development of different postoperative complications compared with those with degenerative diseases [5–7]. Different complications have various adverse impacts on surgery outcomes and patients' postoperative prognosis. According to the Clavien–Dindo classification, postoperative complication severity can be effectively graded for research purposes [8]. Our previous study found that most of the postoperative complications were mild and did not need to be treated and that only severe complications required active treatment. It is of great significance to predict severe postoperative complications in STB patients [9]. To date, research on postoperative complications of STB has been confined to specific complications, such as nerve injury and postoperative intestinal obstruction [10, 11]. Few reports focus on the severity of different postoperative complications. To reduce the risk of serious postoperative complications and enhance the effects of both debridement surgery and postoperative recovery in patients with STB, it is necessary to identify the independent risk factors that affect the severity of postoperative complications in STB.

This study retrospectively examined the data of patients with STB who underwent debridement surgery at the First Affiliated Hospital of Chongqing Medical University to identify the risk factors of different degrees of severity that predict postoperative complications.

## 2. Materials and Methods

All participants provided written informed consent.

### 2.1. Patient Selection

A total of 188 patients with STB who underwent lesion debridement in our hospital between January 2012 and May 2021 were retrospectively included in this study.

The article "Value of Postoperative Serum Albumin to Predict Postoperative Complication Severity in Spinal Tuberculosis" was published in 2022. Journal: Biomed Res Int.

#### 2.1.1. Inclusion Criteria

Patients were selected if they met the following inclusion criteria: (1) medical records were complete, including data on general information, perioperative laboratory examination, imaging results (including magnetic resonance imaging (MRI) and computed tomography (CT)), and clinical data on postoperative complications; (2) patients underwent debridement, bone graft, and instrumented fusion; and (3) lesion tissues were extracted during the surgery, and postoperative pathological diagnosis was confirmed as STB.

#### 2.1.2. Exclusion Criteria

Patients were excluded if they presented with the following: (1) suspected STB not confirmed by pathological examination, (2) preliminary and pathological diagnosis of diseases other than STB, (3) patients without postoperative complication, or (4) a previous history of STB.

### 2.2. Measures and Statistics

#### 2.2.1. Measures

Based on previous studies and our experience, the following possible items for the analysis of different postoperative CDC complications in patients with STB were assessed: patients' preoperative general conditions, surgery-related indicators, and postoperative laboratory indexes. Measures of preoperative general patient conditions included age, sex, body mass index (BMI), comorbidities of diabetes mellitus and pulmonary tuberculosis, history of alcohol use, history of smoking, course of disease, preoperative hemoglobin, preoperative serum albumin, preoperative lymphocytes, preoperative erythrocyte sedimentation rate (ESR), and preoperative C-reactive protein (CRP). Surgery-related indicators included surgical approach, operating time, and blood loss during surgery. Postoperative laboratory indexes included postoperative hemoglobin and postoperative serum albumin. Postoperative complications were divided into different grades based on the Clavien–Dindo classification (Table 1).

#### 2.2.2. Statistical Analysis

Clinical characteristics were assessed using univariate ordinal logistic regression analysis, and significant factors with *P* < 0.1 were entered into a multivariate ordinal logistic regression. ROC curve analysis determined the threshold values for continuous variables. *P* < 0.05 was considered as indicating statistical significance. SPSS version 26.0 software was used for statistical analyses.

## 3. Result

### 3.1. Patient Population

In total, 188 patients presented with postoperative complications and were enrolled in the study, including 102 males and 86 females (Figure 1). Patients' various complications are shown in Table 2. Mean ages, BMI, smoking and alcohol use history, and disease course of patients in the three groups are shown in Figure 1. Operation time, operation blood loss, surgery approach, postoperative hemoglobin, and postoperative albumin of patients in the three groups are shown in Figures 2 and 3.

The article "Value of Postoperative Serum Albumin to Predict Postoperative Complication Severity in Spinal Tuberculosis" was published in 2022. Journal: Biomed Res Int.

### 3.2. Results of Univariate and Multivariate Ordinal Logistic Regression Analyses

Univariate ordinal logistic regression analysis showed that sex, diabetes mellitus, postoperative hemoglobin, and postoperative serum albumin were all risk factors for the severity of different postoperative Clavien–Dindo complications (Table 3). Multivariate ordinal logistic regression analysis of the above significant risk factors revealed that postoperative serum albumin was an independent risk factor for postoperative complication severity (Table 4).

### 3.3. ROC Curve Analysis

ROC curves showed that the diagnostic thresholds of postoperative serum albumin in CDC II and CDC III-IV were 32 g/L (sensitivity: 0.571, specificity: 0.714, area under the ROC curve: 0.680) and 30 g/L (sensitivity: 0.649, specificity: 0.800, area under the ROC curve: 0.697), respectively (Figure 4).

## 4. Discussion

In the present study, ordinal logistic regression analysis revealed that postoperative serum albumin level was an independent risk factor for postoperative complication severity in patients with STB.

Serum albumin is a plasma protein synthesized by the liver, which plays an important role in maintaining blood colloid osmotic pressure and transporting metabolic substances. As an endogenous nutrient, albumin is the most commonly used and most reliable evaluation index for the body's nutritional status [12–14]. Preoperative malnutrition is common in patients with STB, and it has been reported that between 4.8% and 16.8% of patients who underwent spinal surgery develop preoperative hypoalbuminemia as a complication [15, 16]. STB is considered a chronic wasting disease, and patients with STB have a higher risk of preoperative hypoalbuminemia. After STB surgery, patients have significantly reduced levels of postoperative albumin, and in one study, the incidence of postoperative hypoalbuminemia has been found to be 72.8% [17]. Many factors can lead to low albumin levels, including insufficient protein intake or malabsorption, protein synthesis disorder, increased albumin catabolism rate, abnormal albumin distribution, and external albumin loss [18–21]. There are two main factors that lead to low albumin levels in patients with STB. First, STB is a chronic wasting disease with 25.7% of patients experiencing pulmonary tuberculosis as a complication. These patients have high nutritional requirements and lower protein intake, and the inflammation caused by the tuberculosis infection increases albumin consumption, which in turn leads to the half-life time of albumin being decreased to 8.2 ± 1.4 days, while the normal value is 12.5 ± 1.7 days [22, 23]. Second, debridement surgery in patients with STB is a critical factor that can lead to low postoperative albumin levels. Compared with surgery for degenerative spinal disease, STB surgery also involves focus debridement as a step, resulting in longer operating time, more bleeding, and more trauma. Surgery has several effects on postoperative albumin levels. (a) First, bleeding following surgery removes some of the albumin from the blood and dilutes the remaining serum albumin concentration [24]. (b) Second, surgery leads to a physiological stress state and inflammatory reaction, which injures the capillary endothelial cells in the whole body and increases capillary permeability. Thus, the albumin in the blood vessel penetrates into the tissue space and reduces serum albumin, a mechanism called transcapillary escape of albumin [25]. (c) Finally, during this stress state, the liver decreases albumin synthesis and prioritizes acute phase protein synthesis including that of C-reactive protein. Several causes contribute to impaired liver function and reduce the liver's ability to synthesize albumin, which in turn decreases serum albumin [26]. Due to the nature of the disease and the surgical methods used, patients with STB experience significant decreases in serum albumin and are at high risk of hypoalbuminemia following surgery.

The article "Value of Postoperative Serum Albumin to Predict Postoperative Complication Severity in Spinal Tuberculosis" was published in 2022. Journal: Biomed Res Int.

To date, many studies found that preoperative albumin is associated with postoperative complications. Yi et al. found an increased risk of major perioperative complications after total hip replacement in patients with serum albumin levels < 35 g/L [27, 28]. Patients with preoperative hypoalbuminemia have a significantly increased risk of sepsis, myocardial infarction, and perioperative pneumonia after total hip replacement [29, 30]. Patients who underwent cervical surgery with hypoalbuminemia had a higher rate of any major postoperative complications, particularly pulmonary and cardiac complications, and were more likely to require a reoperation and longer hospital stays [31]. Preoperative hypoalbuminemia is a risk factor for postoperative surgical site infection after spinal surgery and prolongs the hospital stay [16, 32]. One of our previous studies also suggested that preoperative albumin is an independent risk factor for overall postoperative complications of STB [33]. Many studies have confirmed that preoperative albumin is significantly associated with postoperative complications in patients with STB. Our study further revealed that postoperative albumin is an independent risk factor for the severity of postoperative complications in patients with STB, and the lower the postoperative albumin, the greater the risk of more serious complications. In addition, when the postoperative albumin is less than 30 g/L, more attention should be paid to the occurrence of complications above CDC III grade. Such complications have important implications for perioperative management and enhanced recovery after surgery of patients and indicate that clinicians should pay more attention to postoperative albumin levels in patients with STB.

The article "Value of Postoperative Serum Albumin to Predict Postoperative Complication Severity in Spinal Tuberculosis" was published in 2022. Journal: Biomed Res Int.

It remains controversial whether exogenous albumin supplementation should be used to treat postoperative hypoalbuminemia in patients with STB. Exogenous human serum albumin supplementation can effectively improve postoperative albumin levels for patients with hypoalbuminemia after surgery. However, studies have demonstrated that the use of albumin after surgery will not reduce the risk of postoperative incision complications and will increase the risk of postoperative infection [9]. After the infusion of exogenous albumin, about 10% of albumin exudes from the blood vessels within 2 hours, and 75% is distributed outside the blood vessels within 2 days. Also, albumin takes a long time to decompose, and if it cannot decompose, it produces the required amino acids in the short term [18, 34]. In addition, exogenous albumin contains different kinds of amino acids excluding tryptophan and isoleucine and has low nutritional value, and therefore, it is generally not recommended for improving nutritional status and correcting hypoproteinemia [35].

One of our unpublished studies found that albumin in patients with STB decreased every day starting on the first postoperative day, reached the lowest value on the third day, then rose slowly, and returned to a normal level on about the fifth day. The latter may be related to the relief of patients' stress levels following surgery and the release of albumin return from tissues into the blood [24]. Most complications in patients occurred within a week after the application of exogenous albumin. It only took a short time to increase albumin levels to more than 32 g/L. Moreover, the risk of CDC II and higher complications provides guidance for postoperative albumin applications and suggests directions of further research. Most of the complications in patients occur during the first week after surgery. If exogenous albumin is applied for a short time within one week after surgery and the albumin level is increased to more than 32 g/L, the risk of CDC II level complications may be reduced. This in turn may provide further guidance for the application of albumin after surgery and for further research.

The article "Value of Postoperative Serum Albumin to Predict Postoperative Complication Severity in Spinal Tuberculosis" was published in 2022. Journal: Biomed Res Int.

## 5. Conclusion

This investigation identified postoperative albumin as an independent risk factor for the severity of postoperative complications in patients with STB. When postoperative albumin was less than 32 g/L, there is a high risk of occurrence of CDC II complications, and when postoperative albumin is less than 30 g/L, CDC III-IV complications have a high risk of incidence occurrence. The improvement of postoperative albumin levels may reduce the risk of severe complications in patients with STB.

## 6. Study Limitations

This study has some limitations. First, there may be some risk factors we did not take into inclusion. Second, a better complication classification method may exist. Third, a larger sample size would increase the statistical power available and hence the ability to detect smaller effect sizes. Fourth, this study is a retrospective study; the role of improvement of postoperative albumin in complication prevention needs to be evaluated. Future studies addressing these limitations will be required to confirm these results.

## Figures and Tables

**Figure 1:** Preoperative clinical characteristic comparisons of grade I, grade II, and grade III–IV complication groups using the Clavien–Dindo classification.

**Figure 2:** Comparisons of surgery-related clinical characteristics of grade I, grade II, and grade III–IV complication groups using the Clavien–Dindo classification.

**Figure 3:** Postoperative clinical characteristic comparisons of grade I, grade II, and grade III–IV complication groups using the Clavien–Dindo classification.

**Figure 4:** Receiver operating characteristic curves of postoperative serum albumin for grade II and grade III-IV complications.

**Table 1:** Details of the Clavien–Dindo classification of complications.

Grade	Definition
I	Any deviation from the normal postoperative course without the need for pharmacological treatment or surgical, endoscopic, and radiological interventions; allowed regimens are antiemetics, antipyretics, analgesics, diuretics, electrolytes, and physiotherapy; includes wound opened at the bedside
II	Requiring pharmacological treatment with drugs other than those allowed for grade I; includes blood transfusions and total parental nutrition
III	Requiring surgical, endoscopic, or radiological intervention
IIIa	Intervention not under general anesthesia
IIIb	Intervention under general anesthesia
IV	Life-threatening complication requiring intensive care unit management
IVa	Single organ dysfunction (including dialysis)
IVb	Multiorgan dysfunction
V	Death

**Table 2:** Details of patients with the Clavien–Dindo classification of complications.

	Number
Total	188
Clavien–Dindo I	77 (41.0%)
Low serum albumin	58
Mild and moderate anemia	61
High fever	28
Gastrointestinal symptoms	25
Cerebrospinal fluid leakage	9
Electrolyte disorders	10
Clavien–Dindo II	91 (48.4%)
Hypoalbuminemia	41
Severe anemia	11
Abnormal liver function	18
Abnormal kidney function	4
Delirium	2
Limb nerve symptoms	14
Drug side effect	8
Thrombus	3
Urinary tract infection	2
Clavien–Dindo IIIa	12 (6.4%)
Wound infection and/or poor healing	11
Restricted respiratory function	1
Clavien–Dindo IIIb	7 (3.7%)
Pleural effusion	5
Rupture of iliac vein	1
Internal fixation instability	1
Clavien–Dindo IVa	1 (0.5%)
Respiratory failure	1

The article "Value of Postoperative Serum Albumin to Predict Postoperative Complication Severity in Spinal Tuberculosis" was published in 2022. Journal: Biomed Res Int.

**Table 3:** Univariate ordinal logistic regression analysis of risk factors in patients with different grades of complications.

Characteristics	Estimate (SE)	Unadjusted odds ratio (OR)	95% CI	*P* value
Age	0.012	1.012	-0.005-0.029	0.178
Sex	-0.623	0.536	-1.181-0.065	0.029^∗^
BMI	-0.036	0.965	-0.117-0.046	0.391
Diabetes mellitus	-0.684	0.505	-1.414-0.047	0.066^∗^
Pulmonary tuberculosis	-0.271	0.763	-0.827-0.286	0.340
Smoking history	-0.007	0.993	-0.027-0.013	0.515
Alcohol use history	0.000	1.000	-0.025-0.025	0.984
Course of disease	0.001	1.001	-0.008-0.011	0.754
Preoperative hemoglobin	0.013	1.014	0.983-1.045	0.388
Preoperative serum albumin	-0.025	0.975	-0.092-0.041	0.458
Preoperative lymphocytes	-0.101	0.904	-0.724-0.523	0.751
Preoperative CRP	0.000	1.000	-0.008-0.008	0.910
Preoperative ESR	0.005	1.005	-0.005-0.016	0.323
Surgery approach	0.020	1.020	-0.833-0.872	0.964
Operating time	0.003	1.003	-0.002-0.007	0.319
Blood loss during surgery	0.000	1.000	-0.001-0.001	0.463
Postoperative hemoglobin	-0.034	0.967	-0.055-0.014	0.001^∗^
Postoperative serum albumin	-0.169	0.845	-0.241-0.096	<0.001^∗^

BMI: body mass index; CRP: C-reactive protein; ESR: erythrocyte sedimentation rate.

**Table 4:** Multivariate ordinal logistic regression analysis of risk factors in patients with different grades of complications.

Characteristics	Estimate (SE)	Crude odds ratio (OR)	95% CI	*P* value
Sex	-0.435	0.647	-1.051-0.180	0.166
Diabetes mellitus	-0.358	0.699	-1.117-0.401	0.355
Postoperative hemoglobin	-0.011	0.989	-0.036-0.014	0.396
Postoperative serum albumin	-0.150	0.861	-0.230-0.069	<0.001^∗^

## Data Availability

The data used to support the findings of this study are available from the corresponding author upon request.
